# Management practice, and adherence and its contributing factors among patients with chronic kidney disease at Tikur Anbessa Specialized Hospital: A hospital-based cross-sectional study

**DOI:** 10.1371/journal.pone.0200415

**Published:** 2018-07-25

**Authors:** Belayneh Kefale, Yewondwossen Tadesse, Minyahil Alebachew, Ephrem Engidawork

**Affiliations:** 1 Department of Pharmacy, College of Medicine and Health Science, Ambo University, Ambo, Ethiopia; 2 Department of Internal Medicine, School of Medicine, College of Health Sciences, Addis Ababa University, Addis Ababa, Ethiopia; 3 Department of Pharmacology and Clinical Pharmacy, School of Pharmacy, College of Health Sciences, Addis Ababa University, Addis Ababa, Ethiopia; Srinakharinwirot University, THAILAND

## Abstract

**Introduction:**

Chronic kidney disease (CKD) has a complicated interrelationship with other diseases and major risk factor for cardiovascular disease. Therapeutic management for CKD patients is complicated due to co-morbidities and dominant risk factors of CKD. Non-adherence to treatment is an increasing problem for patients with CKD and it has not been extensively studied in patients with CKD. Hence, the present study was carried out to assess the management practice, medication adherence and factors affecting medication adherence in CKD patients at Tikur Anbessa Specialized Hospital (TASH).

**Methods:**

A hospital-based cross-sectional study was conducted at the nephrology clinic of TASH. A total of 256 patients were recruited through systematic random sampling. Data were collected from medical records and interviewing patients. The degree of adherence was determined using eight-item Morisky Medication Adherence Scale. The data were entered into Epi Info 7.2.2.2 and analyzed using SPSS version 20.0 statistical software. Descriptive statistics such as frequency, percent, mean and standard deviation were used to summarize patients’ baseline characteristics. Univariable and multivariable binary logistic regression were used to investigate the potential predictors of medication non-adherence.

**Results:**

About 55% patients with hypertension only were treated with non-angiotensin converting enzyme inhibition based regimens; 57.3% of diabetes mellitus with hypertension treated with combination of insulin and ACEI based regimens. About three-fourth of patients with anemia and osteodystrophy complications were treated with iron preparations and calcium based phosphate binder. Only 61.3% of the study population were adherent to their treatment regimens. Forgetfulness (79.8%) was the major reason for medication non-adherence. Patients who had an average and high monthly income were 4.14 (AOR = 4.14, 95% CI: 1.45–11.84, p = 0.008) and 6.17 times (AOR = 6.17, 95% CI: 1.02–37.46, p = 0.048) more likely to adhere as compared to those who had very low income. Patients who were prescribed with ≥5 drugs were 0.46 times (AOR = 0.54, 95% CI: 0.27–1.10, p = 0.049) less likely to adhere compared to their counterpart. Patients who were students, drivers, teachers working in private school were about 7.46 times (AOR = 7.46, 95% CI: 1.49–37.26, p = 0.014) more likely to adhere compared with patients who were farmers.

**Conclusion:**

Insulin and ACEIs based regimens were the most frequently used regimens in the treatment of diabetes mellitus and hypertension co-morbidities. Very low income, increased number of prescribed medications and being a farmer were the predictors of medication non-adherence.

## Introduction

Chronic kidney disease (CKD) is defined as abnormal kidney structure or function persisting greater than 3 months [1]. It is a progressive, irreversible deterioration in renal function in which the body’s ability to sustain metabolic and fluid and electrolyte balance fails, resulting in uremia or azotemia [2]. Increasing prevalence of declining renal function, diabetes, hypertension, primary renal disorders, glomerulonephritis and obesity [3, 4] has contributed to CKD becoming one of the most common chronic diseases [5].

CKD has a complicated interrelationship with other diseases, most commonly diabetes mellitus, hypertension and glomerulonephritis [6]. It is a global public health problem due to the rapid rise of common risk factors such as diabetes and hypertension will result more profound burden that developing nations are not equipped to handle [7]. It is associated with serious consequences, including, increased risk of mortality, accelerated CVD and increased risk of acute kidney injury [1]. Mortality from CVD is estimated to be at least 8 to 10 fold higher in CKD patients as compared to non-CKD patients [7]. Recent studies have reported that CKD is an independent and major risk factor for cardiovascular disease (CVD) [1, 8]. Attention to cardiovascular risk factors remains the cornerstone of management to delay progression of CKD and prevent cardiovascular events. The direct management of CKD focuses on renin angiotensin aldosterone system, blood pressure and glycemic control. Optimal management of common co-morbid conditions and addressing cardiovascular risk factors are important to slow down its progression, reduce the risk of developing CVD for as long as possible [9].

Globally, 10% of the population is affected by CKD, and millions die each year due to high economic cost treatment [1]. It affects 10–15% (western countries) [10], 17.2% (India) [11], 14.82% (China) [12] of the adult population, many of whom require costly treatments. With increasing of aging population, elderly people are the highest risk group for CKD. Studies in US and China population showed that prevalence of CKD (US & China): stage 1 (1.8% & 3.33%), stage 2 (3.2% & 2.49%), stage 3 (7.7% & 7.07%) and stages 4 and 5 (0.35% & 0.97%) [12, 13].

Incidence of the disease increases at an annual rate of 8%, and consumes up to 2% of the total global health expenditure [14]. The treatment of CKD co-morbidities and complications in developing countries is expensive, unaffordable, and unavailable [15]. Suboptimal management of co-morbid conditions and non-adherence to prescribed medication schedule have been the major problems in CKD patients and their occurrence can adversely impact the course of the disease [16, 17]. Non-adherence to treatment regimens is common, leading to considerable deterioration of the disease and enhanced healthcare expenditure. According to World Health Organization, it is estimated that only 50% of people with chronic diseases take their medications consistently as prescribed because they consider them ineffective or experience untoward side effects [18]. The pill burden in CKD patients is high, have to take on average around 8–10 tablets/day, due to the existence of co-morbidities and dominant risk factors of CKD [19]. Hence, CKD patients belong to the group of subjects with one of the highest burdens of daily pill intake depending on severity of their disease [20]. This imposes high personal and economic burden on patients and their families [5, 17, 21].

Though non-adherence to treatment is an increasing problem for patients with CKD, it has not been extensively studied in patients with CKD [22]. Previous studies have reported that 24.8% [23], 26–28% [16], 46.1% [24], 78% [25], 18.4% [26] and 23.8% [27] of CKD patients were non-adherent in California, Brazil, the Netherlands, India, Germany and southern Ethiopia, respectively.

The incidence of CKD in Ethiopia is rising because of increased risk factors [27]. Evidence-based research that evaluates management practice and medication adherence among patients with CKD in developing countries is scanty [28]. Thus, there should be a continuing need to routinely assess management practice, rate of adherence and factors affecting medication adherence among patients with CKD in health facilities [23, 29]. This is particularly imperative in resource-limited countries, as the predominance of economic instability, inadequate follow up, missed appointments and inaccessibility of healthcare facilities might contribute to the incidence of poor medication adherence [30, 31] (Fig 1). Hence, the present study was carried out to assess the management practice, medication adherence and factors affecting adherence in CKD patients at TASH.

**Fig 1:** Structural framework for contributing factors of medication adherence.

## Methods and materials

### Study settings

The study was conducted in the renal ambulatory clinics of TASH, which is located in Addis Ababa, Ethiopia. TASH is the largest general public hospital, where tertiary care is being provided in Ethiopia, with over 800 beds. TASH serves about 500,000 patients per year in its outpatient department and about 40,000 in the inpatient and same number in the emergency department and about 600 adult CKD patients. The renal Clinic has nephrologists, nurses and pharmacists. It provides treatment to different types of renal disease and its complications.

### Study design and period

A hospital-based cross-sectional study was conducted in two-phases. The first was a patient interview phase, while the second was a retrospective patient chart review. The two-phases were done for the same patient from May 1^st^–September 30^th^ 2017 to assess management practice and adherence.

### Sample size and sampling methods

The sample size was calculated using single population proportion formula [32] as follows:

n=Zα22p(1−p)d2

Where;

𝑛 = is desired sample size for population >10,000;

Z = is standard normal distribution usually set as 1.96 (which corresponds to 95% confidence level);

P = means that we use positive prevalence estimated, to maximize sample size. Negative prevalence = 1 − 0.5 = 0.5,

d = degree of accuracy desired (marginal error is 0.05); then the sample size is

$$n=\frac{1.96^{2}0.5(1-0.5)}{{\left(0.05\right)}^{2}}=384.18=∼384$$

The expected number of source population in the study period (N), based on the average number of patients coming to the clinic three days in a week with a total of 20 weeks was 600 (20*6+20*12+20*12). The corrected sample size, using the following correction formula was 233.1 ∼ 233,

$$\mathrm{Corrected}\;\mathrm{sample}\;\mathrm{size}=\frac{n\times N}{n+N}$$

Then 10% contingency was added on 233:

233x10%=23

$$233+\mathrm{contingency}=Nf=\underline{256}$$

A systematic random sampling method was used to recruit samples for the study in each day of the data collection process. The actual sampling fraction (k) varied in the different days of data collection as the total number of study population varied in different days. Hence, it was calculated through dividing the number of study population available each day by the maximum possible number of patients’ that could be interviewed the same day. Then, every k^th^ patient was interviewed after physician visit.

### Inclusion and exclusion criteria

#### Inclusion criteria

- All CKD ambulatory patients and on medications for more than 6 months;
- ≥18 years of age

#### Exclusion criteria

- Patients refused to participate in the study
- Patients with cognitive impairment.

### Data collection and analysis

#### Instruments

Data were collected using structured questionnaire and data abstraction format to extract information from the patients and medical records, respectively (S1 Annex). The questionnaire for the interview contained socio-demographic characteristics, 8-item Morisky Medication Adherence Scale (MMAS-8), which is a validated scale, was utilized to collect information necessary to assess medication adherence and reasons contributing for non-adherence. MMAS-8 is part of the World Health Organization case management adherence guideline assessment tools and mostly used to classify patients on medication as ‘poor’(a patient who scored <6 for the MMAS-8), ‘moderate’(a patient who scored <8 and >6 for the MMAS-8), and ‘high’ (a patient who scored 8 for the MMAS-8) on motivation and knowledge domain, thus a commonly used self-report method to assess patients’ adherence to existing therapy. MMAS-8 is a 7 items with yes/no response options and 1 item with a 5-point likert scale response option.

In addition, data abstraction format was prepared to extract information such as, management practices and clinical parameters.

#### Data collector’s recruitment and training

Three nurses were recruited as data collectors. Training was given to them regarding appropriate use of the data collection instruments focusing on uniform interpretation of questions, strict use of study criterion, explanation of study objectives and getting verbal consents from study participants, implementation of sampling technique and confidentiality of the collected data.

#### Data quality control

The data collection instrument which consisted of the questionnaire and the data abstraction format was assessed by an expert physician in the field of nephrology for clarity and comprehensiveness of its contents. Pre-testing was done on 5% of the study participants before the start of the actual study. All the necessary modifications and adjustments were done before implementing in the main study.

#### Data analysis and interpretation

Data were sorted, cleaned, coded and entered into SPSS version-20.0 statistical software for management and analysis. Descriptive statistics were used to summarize patients’ baseline characteristics. Bivariate analysis was conducted to see the existence of association between adherence and independent variables. All variables with p<0.2 in the bivariate analysis were included in the multivariable binary logistic regression, which was performed to determine the potential predictors of non-adherence. Adjusted Odds Ratio (AOR) with its p-value and confidence interval (95%) was reported in each logistic regression analysis. P-value < 0.05 considered as statistically significant.

### Ethical consideration

Ethical clearance and approval of the study protocols was obtained from the Ethical Review Board of School of Pharmacy, Addis Ababa University. In addition, permission was sought from the respective heads of Department of Internal Medicine and renal clinic to conduct the study in the clinic. Prior to data collection, individuals were informed about the study and verbal consent was obtained from the study participants. An audio recording made, which was approved by Ethical Review Board of School of Pharmacy. Each patient was informed about the objective of the study, procedures of selection and assurance of confidentiality and their right to refuse was maintained. No identifiers were used to minimize social desirability bias and enhance anonymity.

## Results

### Socio-demographic characteristics

Males comprised 58% of the sex category. Majority of the participants were in the age group of less than 61 years, which accounted for 54.3%. Mean age of the study population was 52.5 (SD = 16.8) years (range 18 to 90 years). Married participants accounted for 69.9% and being retired (25.4%) and government employee (23.4%) accounted for the highest percentage of occupation. Education-wise, 34.4% and 27.7% attended primary and higher education, respectively. Majority of the participants were non-health professionals (97.3%). A significant proportion of the study participants (29.7%) had low level of monthly family income (Table 1).

**Table 1:** Socio-demographic characteristic of chronic kidney disease patients attending the renal clinic of Tikur Anbessa Specialized Hospital.

Variables	Stage of CKD				
	1 & 2 (n = 50)	3 (n = 88)	4 (n = 55)	5 (n = 63)	Total (n = 256)
**Sex**					
Male	25 (50)	60 (68.2)	31 (56.4)	33 (52.4)	149 (58)
Female	25 (50)	28 (31.2)	24 (43.6)	30 (47.6)	107 (42)
**Age (years)**					
≤60	38 (76)	41 (46.6)	28(50.9)	32(50.8)	139 (54.3)
>60	12(24)	47 (53.4)	27(49.1)	31(49.2)	117 (45.7)
**Marital status**					
Singleς	14(28)	23(26.1)	20(36.4)	20(31.7)	77 (30.1)
Married	36(72)	65(73.9)	35(63.6)	43(68.3)	179 (69.9)
**Occupation**					
Farmer	6(12)	8(9.1)	4(7.3)	6(9.5)	24 (9.4)
Gov’t employee	18(36)	19(25.6)	11(20)	12(19.1)	60 (23.4)
Merchant/trade	7(14)	5(5.7)	5(9.1)	6(9.5)	23 (9)
Daily laborer	2(4)	6(6.8)	4(7.3)	7(11.1)	19 (7.4)
House wife	7(14)	11(12.5)	8(14.5)	11(17.5)	37 (14.5)
Retired	6(12)	27(30.7)	18(32.7)	14(22.2)	65 (25.4)
Others*	4(8)	12(13.6)	5(9.1)	7(11.1)	28 (10.9)
**Profession**					
Health professional	3(6)	1(1.1)	2(3.6)	1(1.6)	7 (2.7)
Non-health professional	47(94)	87(98.9)	53(96.4)	62(98.4)	249 (97.3)
**Educational status**					
Cannot read and write	5(10)	11(12.5)	7(12.7)	7(11.1)	30 (11.7)
Primary	13(26)	31(35.23)	20(36.4)	24(38.1)	88 (34.4)
Secondary	10(20)	23(26.1)	19(34.5)	15(23.8)	67 (26.2)
Higher Education	22(44)	23(26.1)	9(16.4)	17(27)	71 (27.7)
Monthly family income (ETB)**					
Very low (≤860)	4(8)	10(11.4)	11(20)	15(23.8)	40 (15.6)
Low (861–1500)	13(26)	21(23.9)	17(30.9)	21(33.3)	72 (28.1)
Average (1501–3000)	10(20)	33(37.5)	18(32.7)	15(23.8)	76 (29.7)
Above average (3001– 5000)	17(34)	20(22.7)	6(10.9)	8(12.7)	51 (19.9)
High (≥5001)	6(12)	4(4.5)	3(5.5)	4(6.4)	17 (6.7)

ςSingle, divorced and widowed

*students, driver, garage (mechanic), guard, teacher working in private school

** Based on the Ethiopian Civil Service monthly salary scale for civil servants

### Disease related characteristics

Overall, patients had been diagnosed with CKD for an average of 4.7 (SD = 3.5) years, ranging from under five years (158, 61.7%) through 5–10 years (75, 29.3%) to above ten years (23, 9%) (Fig 2).

**Fig 2:** Duration of chronic kidney disease among patients attending the renal clinic of Tikur Anbessa Specialized Hospital.

About two-third (64.4%) of the study participants did not have long term complications. Cardiovascular disease and anemia accounted for the highest percentage among patients that had at least one long term CKD complications. Almost all (96.5%) patients had at least one co-morbid condition, hypertension being the major type of co-morbidity (91.1%) (Table 2).

**Table 2:** Presence of co-morbidities and complications among chronic kidney disease patients attending the renal clinic of Tikur Anbessa Specialized Hospital.

Variables	Frequency	Percent
**Co-morbidities**		
Absent	9	3.5
Present	247	96.5
**Specific Co-morbidities (n = 247)**		
Hypertension	225	91.1
Diabetes mellitus	114	46.2
Ischemic Heart Disease	33	13.4
Dyslipidemia	31	12.6
Stroke	10	4.1
Others*	22	13
**Complications**		
Absent	165	64.4
Present	91	35.6
**Specific complications (n = 91)**		
Cardiovascular disease	29	31.9
Anemia	28	30.8
Osteodystrophy	23	25.2
Edema	14	15.3
Hyperkalemia	10	11
Peripheral neuropathy	9	9.9

*Gouty arthritis, asthma, Parkinson, nephritic syndrome, pyelonephritis

### Non-pharmacological management approaches

The present study revealed that diet restriction, exercise and no-smoking were the most commonly used non-pharmacological approaches. Agreed dietary plan was found to be present in most (68.8%) of the patients (Table 3).

**Table 3:** Non-pharmacological management approaches used among chronic kidney disease patients attending the renal clinic of Tikur Anbessa Specialized Hospital.

Variables	Frequency	Percent
**Dietary Approach**		
Presence of agreed dietary plan with physician		
Yes	175	68.4
No	81	31.6
Salt restriction (n = 175)		
Yes	167	95.4
No	8	4.6
Cut off sweet carbohydrate meals (n = 114)	114	100
**Exercise**		
Presence of agreed exercise plan with physicians		
Yes	130	50.8
No	126	49.2
Exercising according to plan (n = 130)		
Yes	120	92.3
No	10	7.7
Days per week doing moderate intense exercise		
< 3 Days	7	5.4
≥3 Days	123	94.6
Duration of moderate intense exercise per week in minutes		
< 140 Minutes	64	49.2
≥140 Minutes	66	50.8
**Cigarette**		
Ever smoked		
Yes	28	10.9
No	228	89.1
Smoking now (n = 28)		
Yes	4	14.3
No	24	85.7

#### Profile of prescribed medications

Table 4 presents medication profile of patients based on CKD stages. It revealed that enalapril (133, 52%) was the most commonly prescribed drug followed by furosemide (128, 50%) and amlodipine (124, 48.4%). Insulin and ASA (Acetyl Salicylic Acid) were found to be the major type of antidiabetic and cardiovascular medications which were prescribed for 69 (27%) and 70 (27.3%) patients, respectively. The average number of prescribed drugs per patient was 3.9 (SD = 2.2) with a range of 0–12 drugs (Table 4).

**Table 4:** Profile of prescribed medications for chronic kidney disease patients attending the renal clinic of Tikur Anbessa Specialized Hospital.

Variables	Number of medications prescribed across CKD stages per patient				
	1 & 2 (n = 50)	3 (n = 88)	4 (n = 55)	5 (n = 63)	Total (n = 256)
**Angiotensin converting enzyme inhibitors**					
Enalapril	41 (82)	47 (53.4)	32(58.2)	28(44.4)	148 (57.8)
**Calcium channal blockers**					
Amlodipine	21(42)	41(46.6)	25(45.5)	37(58.7)	124 (48.4)
Nifedipine	8(16)	13(14.8)	17(30.9)	13(20.6)	51 (19.9)
**Diuretics**					
Furosemide	14(28)	38(43.2)	30(54.5)	46(73)	128 (50)
Hydrochlorothiazide	10(20)	23(26.1)	14(24.5)	22(34.9)	69 (27)
Spironolactone	4(8)	12(13.6)	4(7.3)	10(15.9)	30 (11.7)
**β-blocker**					
Atenolol	6(12)	13(14.8)	10(18.2)	20(31.7)	49 (19.1)
Metoprolol	4(8)	5(5.7)	3(5.5)	1(1.6)	13 (5.1)
Carvedilol	0(0)	4(4.5)	1(1.8)	2(3.2)	7 (2.74)
**Angiotensin receptor blockers**					
Losartan	1(2)	2(2.3)	2(3.6)	0(0)	5(2)
**Antidiabetic Medications**					
Insulin	14(28)	14(15.9)	20(36.4)	21(33.3)	69 (27)
Metformin	9(18)	8(9.1)	4(7.3)	5(7.9)	26 (10.2)
Glibenclamide	1(2)	5(5.7)	2(3.6)	0(0)	8 (3.1)
**Other medications**					
Acetyl salicylic acid	8(16)	23(26.1)	20(36.4)	19(30.2)	70 (27.3)
Statins	9(18)	18(20.5)	8(14.5)	15(23.8)	50 (19.5)
Calcium based phosphate binder	1(2)	3(3.4)	6(10.9)	15(23.8)	25 (9.8)
Iron	0(0)	4(4.5)	9(16.4)	15(23.8)	28 (10.9)
Antibiotics	1(2)	5(5.7)	5(9.1)	5(7.9)	16 (6.3)
Others*	15(30)	23(26.1)	13(23.6)	17(27)	68 (26.6)
**Number of medications**	3.2 ± 1.6	3.5 ± 1.7	4.3 ± 2	4.9 ± 2.9	3.9 ± 2.2

* Phenobarbitone, Warfarin, Prednisolone, Antiretroviral therapy, Carbamazepine, Chlorpromazine

#### Management practice for co-morbidities and complications

Respondents were placed on different medications for treatment of CKD co-morbidities or complications. Hypertension was managed by combination of drugs, non-ACEI based (55%) being the most commonly used combination followed by ACEI based (45%). Insulin and metformin were the most commonly prescribed drugs in the management of diabetes mellitus alone. In diabetes mellitus and hypertension co-morbidities, insulin and ACEI based combinations (57.3%) and ACEI based combinations (19.8%) were the two most commonly used combinations (Table 5).

**Table 5:** Types of regimens used in the management of chronic kidney disease co-morbidities patients attending the renal clinic of Tikur Anbessa Specialized Hospital.

Co morbidities	Frequency	Percent (%)
**Hypertension (n = 129)**		
Angiotensin converting enzyme inhibitors based regimens	58	45
Non-ACEI based regimens	71	55
**Diabetes mellitus + hypertension (n = 96)**		
Insulin + Angiotensin converting enzyme inhibitors based regimens	55	57.3
Angiotensin converting enzyme inhibitors based regimens	19	19.8
Metformin + Angiotensin converting enzyme inhibitors based regimens	13	13.5
Insulin + Non- Angiotensin converting enzyme inhibitors based regimens	5	5.2
Metformin + Non- Angiotensin converting enzyme inhibitors based regimens	4	4.2
**Diabetes Mellitus (n = 18)**		
Insulin	8	44.4
Metformin	6	33.3
Glibenclamide	3	16.7
Insulin + Glibenclamide	1	5.6
**Ischemic heart disease (n = 33)**		
Acetyl salicylic acid + β-Blocker	33	100
**Dyslipidemia (n = 31)**		
Statins	31	100
**Stroke (n = 10)**		
Acetyl salicylic acid	10	100
Others* **(n = 12)**		
Acetyl salicylic acid + others^ς^	7	58.3
Statins + others^ς^	5	41.7

*Asthma, HIV/AIDS, gout, nephritic syndrome

^ς^Phenobarbitone, antibiotics, prednisolone, antiretroviral therapy, carbamezapine.

#### Types of regimens used in the management of complications of chronic kidney disease

ACEIs alone (18%) or in combination (52%) were the most commonly prescribed agent for treating CVD related complications. About three-fourth of anemia & osteodystrophy were treated with iron preparation & calcium based phosphate binder, respectively. Likewise, 92.3% of edema, 40% of hyperkalemia and 88.9% of peripheral neuropathy were treated with furosemide, calcium gluconate and amitriptylin, respectively (Fig 3).

**Fig 3:** Management practice of complications among chronic kidney disease patients attending the renal clinic of Tikur Anbessa Specialized Hospital.

### Rate of adherence and reasons for non-adherence

Assessment of patients’ responses to the 8-item Morisky Medication Adherence Scale showed that 157(61.3%), 51(19.9%) and 48(18.8%) patients exhibited high, medium and poor adherence to the prescribed regimens, respectively (Fig 4).

**Fig 4:** Rate of adherence to medications among chronic kidney disease patients in renal clinic of Tikur Anbessa Specialized Hospital.

Upon evaluation of the reasons for CKD medication non-adherence, it was identified that forgetfulness (79.8%) was the main reason for their non-adherence. Furthermore, side effects of the medications and high cost of medications accounted for 49.5% and 38.4% of medication non-adherence, respectively. Feeling well without treatment and physicians’ mode of approach were, however, the least common reasons for non-adherence (Fig 5).

**Fig 5:** Reasons for medication non-adherence among chronic kidney disease patients attending the renal clinic of Tikur Anbessa Specialized Hospital.

#### Factors associated with medication adherence

Based on the results of univariate binary logistic regression analysis, variables such as sex, age, occupation, educational status, family income, CKD stage, number of medications and co-morbidities were included in the multivariate logistic regression analysis. After controlling different demographic, economical and other factors through the use of multivariate logistic regression analysis, this study showed that only family income, total number of prescribed drugs and occupation had significant association with CKD medication adherence. Accordingly, patients who had an average and high family monthly income were about four (AOR = 4.14, 95% CI: 1.45–11.84, p = 0.008) and six (AOR = 6.17, 95% CI: 1.02–37.46, p = 0.048) times, respectively, more likely to adhere as compared to those who had very low income. During a multivariate logistic regression analysis, it was also found that, patients with other groups (students, driver, teacher working in private school) of occupation had a significant association with their adherence condition and were about seven (AOR = 7.46, 95% CI: 1.49–37.26, p = 0.014) times more likely to adhere compared with patients who were farmers. On the other hand, patients who were prescribed with five and above drugs were 0.46 (AOR = 0.54, 95% CI: 0.27–1.10, p = 0.049) times less likely to adhere compared to those prescribed with less than five drugs (Table 6).

**Table 6:** Univariate and multivariate binary logistic regression analysis of predictors of medication non-adherence.

Variables	Adherence		COR, 95% CI	AOR, 95% CI
	Low to moderate adherence	high adherence		
**Sex**				
Female	51	56	1.00	1.00
Male	48	101	1.92(1.15, 3.20)*	1.56(0.76, 3.2)
**Age in years**				
≤60	43	96	1.00	1.00
> 60	56	61	0.49(0.29, 0.81) *	0.64 (0.29, 1.42)
**Occupation**				
Farmer	13	11	1.00	1.00
Gov’t Employee	20	40	2.36(0.90, 6.21)	1.14(0.30, 4.34)
Merchant/Trade	6	17	3.35(0.98, 11.45)	2.99(0.67, 13.36)
Daily Laborer	7	12	2.03(0.59, 6.93)	2.03(0.43, 9.52)
House wife	21	16	0.90(0.32, 2.53)	1.41(0.34, 5.88)
Retired	27	38	1.66(0.65, 4.27)	2.52(0.63, 10.13)
Others*	5	23	5.44(1.55, 19.11)*	7.46(1.49, 37.26)*
**Educational status**				
Cannot read & write	16	14	1.00	1.00
Primary	43	45	1.2(0.52, 2.74)	0.49(0.14, 1.68)
Secondary	24	43	2.05 (0.85, 4.91)	0.69(0.18, 2.69)
Higher Education	16	55	3.93(1.59, 9.74)*	1.14 (0.24, 5.38)
**Family income category**				
Very Low	25	15	1.00	1.00
Low	39	33	1.41(0.64, 3.1)	1.37(0.49, 3.85)
Average	19	57	5.0(2.19, 11.4)**	4.14(1.45, 11.84)*
Above Average	13	38	4.88(1.99, 11.96)**	3.39(0.91, 12.66)
High	3	14	7.78(1.92, 31.59)*	6.17(1.02, 37.46)*
**CKD stage**				
1 & 2	15	35	1.00	1.00
3	23	65	1.21(0.56, 2.61)	1.42(0.58, 3.47)
4	25	30	0.51 (0.23, 1.15)	0.68(0.27, 1.71)
5	36	27	0.32 (0.15, 0.70)*	0.45(0.18, 1.13)
**Number of medications**				
<5	57	120	1.00	1.00
≥ 5	42	37	0.42 (0.24, 0.72)*	0.54 (0.27, 1.10)*
**Number of co-morbidity**				
0–2	75	141	1.00	1.00
≥ 3	24	16	0.36(0.18, 0.71)*	0.85(0.35, 2.11)

COR = crude odd ratio, AOR = adjusted odd ratio

*Statistically Significant at P≤0.05.

**statistically significant at p ≤ 0.001

*students, driver, garage (mechanic), guard, teacher working in private school.

## Discussion

In the present study, different medications were used in the management of co-morbidities and complications of CKD. Enalapril and hydrochlorothiazide were prescribed in 50.8% and 32.7% of CKD stage 4 & 5 patients, although little robust evidence exists on the use of ACEIs in advanced CKD. ACEIs/ARBs increase potassium and decrease GFR [33, 34] and withdrawal of ACEIs/ARBs increase eGFR and hence, delay the onset of renal replacement therapy [35]. Hydrochlorothiazide was used inappropriately in advanced CKD patients, since thiazide diuretics are deemed ineffective [36]. Based on co-morbidity status, non-ACEI based combinations were the most commonly used treatment regimens in the management of hypertension alone. Contrastingly, various clinical guidelines done by Stevens and Levin [37] and Bilo *et al* [38] stated that ARBs or ACEIs are considered as the first line agents in both diabetic and non-diabetic patients with CKD. ARBs or ACEIs are used not only to decrease blood pressure but also slow down the progression of CKD by reducing proteinuria [39, 40]. The KDIGO guideline was commonly used for the management CKD in our setting but they failed to meet. The probable reason for this variation in TASH may be due to the absence of local standard treatment guideline for the management of CKD patients and lack of awarness of physicians practicing in the renal clinic. Besides, it might be due to difficulty in communication between physicians, shortage of multi-disciplinary care team and heavy workload on nephrologists. Coordinated multidisciplinary care team could improve management and outcomes of patients with CKD and essential for the appropriate management of CKD due to associated co-morbidities and complex regimens. Indeed, a systematic review showed that lack of awareness of evidence-based guidelines for CKD results in large variability in the treatment of CKD co-morbidities and complications [41]. A deficiency in the nephrology workforce especially nephrologists for the provision of appropriate management is a critical problem in developing countries [15]. Hence, targeted training for physicians to raise awareness about the management of CKD and development of clinical guidelines should be emphasized.

Regarding the management of diabetes mellitus and hypertension, the present study revealed that combinations of insulin and ACEI based combinations were the most commonly used treatment regimens. This is in agreement with studies done by Levin *et al* [42], Tomson & Baily [43] and Bilo *et al* [38], which stated that ACEIs based combinations were the first line regimens in the management of diabetes mellitus and hypertension co-morbidities in CKD patients. Previous studies demonstrated that if ACEIs were not effective to control BP, then CCB might be added but not used alone since CCBs may lead to albuminuria and greater hyper-filtration [42].

Insulin was the most widely used treatment agent in the management of diabetes alone co-morbidity with CKD at TASH accounting for 44.4%. The finding of this study is comparable with similar studies by Albers *et al* [44] and Dasari *et al* [45], which indicated that renal patients with diabetes suitably managed with insulin. Though, metformin is an inexpensive and effective for type 2 diabetes mellitus there is much concern about the safety of metformin in advanced CKD, particularly the risk of lactic acidosis [45, 46]. Hence, the frequent use of insulin as first line agent may probably be linked to this notion. The risk of metformin induced lactic acidosis will be very high in stage 4–5 CKD patients and hence it is contraindicated in these stages of patients. Accordingly, the use of metformin in this stage was a malplractice in our setting.

In the present study, statins were predominantly used for the treatment of dyslipidemia and reduction of the relative risk of cardiovascular events in CKD patients. Likewise, studies [45] and practice guidelines [47] have shown that statins are routinely used in the treatment of dyslipidemia and reduction of cardiovascular risk. This frequent usage might be due to the superior pharmacological effects of statins to reduce cardiovascular complications as compared to other lipid lowering agents. In addition, statins may have a role in preventing progression of kidney disease and reducing albuminuria [48]. Thus, statins are the standard treatment of choice in the prevention of cardiovascular risks in patients with and without CKD [49]. Furthermore, ASA and β-blocker combinations were predominantly used treatment regimens in ischemic heart disease. This finding is in agreement with a study [45] and practice guideline [47] that reported β-blockers should be initiated for the relief of symptoms and ASA in the primary prevention of cardiovascular events.

Regarding to the management of CKD complications, ACEI based combinations were the most commonly used treatment regimens in cardiovascular complications. This finding is in line with a systematic review that reported ACEIs or ARBs appeared to be the most commonly used regimens to treat heart failure in renal patients [50]. The present study also revealed that iron preparations were predominantly used in the treatment of anemia in CKD patients. Contrastingly, various studies reported the use of erythropoietin stimulating agents with iron preparations were routinely used in the treatment of anemia in renal patients [51]. Hence, the non usage of erythropoietin stimulating agent could probably be due to the financial constraints and limited availability of this agent at TASH. Although Malluche *et al* [52] & Miller [53] demonstrated that the use of calcium-based phosphate binders have been associated with the development of low bone turnover, bone loss, and worsening of vascular calcifications; calcium containing phosphate binders were the most commonly used agents in the management of osteodystrophy at TASH. This could probably be due to the inaccessibility of new non-aluminum, non-calcium (sevelamer hydrochloride and lanthanum carbonate) phosphate binders in this setting, which have lower risk of vascular calcification [54].

Adherence to CKD medications was observed in 61.3% of the study participants. This finding is similar with previous studies conducted in Netherland [24], India [55] & Spain [56] even though the sample size were differ from studies done in Netherland and Spain and different from other studies conducted in Saudi Arabia [20], India [25], German [26], southern Ethiopia [27], Italy [57], United States [58], and Australia [59]. This variation could be attributed to differences in the definition of non-adherence between studies. In addition, methodologies may differ between studies, contributing to variation in the data. For example, direct monitoring methods include drug concentration assays, use of pill markers and direct observation of pill taking, indirect methods include patient self-reports, structured interview, compliance ratings by nurses, prescription refills and pill counts [60].

Prevalence of adherence in the present study was below the recommended level in the literature to attain optimum outcomes [61]. In the light of poor management of CKD co-morbidities and alleged failure of therapeutic regimen, health care providers are urged to measure CKD patients’ treatment adherence. Efforts are needed to increase the medication adherence of these patients so that they could realize the full benefits of prescribed therapies. When accurate and clear information on the importance of medication adherence is provided, patients are encouraged towards self-care and adherence to drug therapy. Healthcare providers should be more cautious towards recognizing adherence problems in order to provide appropriate interventions. Non-adherence to treatment regimen is life-threatening and expensive in renal patients [62], since these patients have various co-comorbidities and prescribed with complex regimens to treat those conditions [63–65]. Various studies reported that medication non-adherence had been associated with increased risk of co-morbidity [66], hospitalization and healthcare expenditure [67].

In this study, multivariate logistic regression analysis showed that total number of prescribed drugs, occupation and family income were found to be significantly associated with CKD medication adherence. As the number of prescribed drugs increased from <5 medication to ≥5 medication, the odds of being adherent was about 0.46 times less and this implies patients with ≥5 medication were found to be less likely to adhere to their medications. Various studies corroborate this finding, as pill burden adversely affects patient adherence to medications. A study done in USA and Italy demonstrated that patients with high pill burden were more likely to be non-adherent [57, 58]. Similar studies also reported that the number of prescribed medications had a significant inverse association with CKD medication adherence [25, 62, 68]. Moreover, occupation had significant association with CKD medication adherence. Patients who were students, drivers, and teachers working in private school were more likely to engage in adherence compared to those who were farmers. This could probably be due to the fact that farmers might be less aware of their disease and the importance of medication adherence when compared with students, driver and teacher working in private school and thus more likely to be more non-adherent.

On the other hand, monthly family income was significantly associated with medication adherence as the family income increased, patients were found to be more likely to adhere to their medications. This finding is in line with previous study, which reported that socioeconomic status had a significant association with medication adherence [69]. A qualitative study done in Australia to explore factors associated with medication adherence in ESRD patients indicated that financial constraints had contributed to medication non-adherence [59]. Income status has been implicated in non-adherence in several studies of renal patients. In addition, low socio-economic status has been significantly associated for medication non-adherence among CKD patients [16]. In developing countries, majority of CKD patients have limited access to health insurance and hence medical care for CKD patients become expensive and subsequently affects their adherence to the treatment regimen. Predominant proportion of CKD patients in developing countries discontinue treatment after initiating dialysis due to financial constraints[70,71].

In this study, patients with poor adherence reported several reasons for not adhering to their medications. The most common reasons were found to be forgetfulness, experiencing side effects, cost and complex regimen. Most of the patients missed their CKD medications due to forgetfulness which is similar with other studies [25, 59]. A qualitative study by Lindberg & Lindberg [72] revealed that forgetfulness and complex regimen due to polypharmacy were identified as the main obstacle for medication adherence.

Treatment success is primary depends on adherence to treatment regimen. Failure to comply with the recommended treatment regimen is detrimental which can affect the quality of life of the patients and the health care system. It can also result in significant worsening of the disease, increased health care expenditure and death. Medication adherence is adversely affected by various factors such as patient centered, therapy related, social and economic, disease and health care system factors. Hence, identification of specific barriers for each patient and designing appropriate preventing strategies are indispensable to mitigate medication adherence [73]. Even though a number of socio-demographic (age, sex & educational status) and clinical characteristics (number of co-morbidities & complications, severity of the disease and laboratory parameters) were found to be significantly associated with non-adherence in various studies [73], in this study were not statistically significant associated. The probable reason for this variation could be due to the sample size and methodological difference. Hence, prospective studies with multiple methods of adherence assessment may be required to identify different factors which affect medication adherence.

## Conclusions

In summary, the present study showed that 55% of hypertensive patients treated with non-ACEI based regimens, which is inappropriate. Insulin and ACEIs based regimens were the most frequently used regimen in the management of diabetes mellitus and hypertension with diabetes co-morbidities. In addition, medication adherence in CKD patients at TASH was found to be suboptimal (61.3%). Forgetfulness was the most important reason preventing optimal adherence to prescribed medications. Socioeconomic status and pill burden had an important role in determining adherence rate to medications. Very low family income, increased number of prescribed drugs and being a farmer were significant predictor of medication non-adherence.

## Supporting information

S1 Annex Structured questionnaire and data abstraction format. (DOCX)

## Abbreviations

ACEI: Angiotensin Converting Enzyme Inhibitor
AOR: Adjusted Odds Ratio
ARB: Angiotensin Receptor Blocker
CCB: Calcium Channel Blocker
CI: Confidence Interval
CKD: Chronic Kidney Disease
COR: Crude Odds Ratio
CVD: Cardiovascular Disease
GFR: Glomerular Filtration Rate
MMAS-8: 8-Item Morisky Medication Adherence Scale
RAAS: Renin Angiotensin Aldosterone System
SPSS: Statistical Package for Social Sciences
TASH: Tikur Anbessa Specialized Hospital
USA: United States of America
